RETRACTED

# Mutant p53 determines pancreatic cancer poor prognosis to pancreatectomy through upregulation of cavin-1 in patients with preoperative serum CA19-9 ≥ 1,000 U/mL

**DOI:** 10.1038/srep19222

**Published:** 2016-01-12

**Authors:** Jin-Feng Xiang, Wen-Quan Wang, Liang Liu, Hua-Xiang Xu, Chun-Tao Wu, Jing-Xuan Yang, Zi-Hao Qi, Ya-Qi Wang, Jin Xu, Chen Liu, Jiang Long, Quan-Xing Ni, Min Li, Xian-Jun Yu

**Affiliations:** 1 Department of Pancreatic and Hepatobiliary Surgery, Fudan University Shanghai Cancer Center, Department of Oncology, Shanghai Medical College, Fudan University; Pancreatic Cancer Institute, Fudan University, Shanghai, China; 2 Department of Medicine, Department of Surgery, the University of Oklahoma Health Sciences Center, Oklahoma City, OK, USA; 3 The Vivian L. Smith Department of Neurosurgery, University of Texas Medical School at Houston, Houston, TX, USA; 4 Fudan University Shanghai Cancer Center, Collaborative Innovation Center for Cancer Medicine, Shanghai, China

## Abstract

Patients with pancreatic ductal adenocarcinoma (PDAC) and preoperative CA19-9 ≥ 1,000 U/mL that does not decrease postresection have the worst prognosis, but the mechanism is unclear. Here, we elucidated the relationship between this signature and driver-gene mutations, and the cavins/caveolin-1 axis. Four major driver-genes (*KRAS, TP53, CDKN2A/p16,* and *SMAD4/DPC4*) that are associated with PDAC and five critical molecules (cavin-1/-2/-3/-4 and caveolin-1) in the cavins/caveolin-1 axis were screened by immunohistochemistry in tumor tissue microarrays. Additionally, six pancreatic cancer cell lines and a spleen subcapsular inoculation nude mouse model were also used. Overexpression of mutant p53 was the major mutational event in patients with the CA19-9 signature. Cavin-1 was also overexpressed, and mutant p53 correlated directly with high cavin-1 expression in pancreatic cancer cell lines and tumor specimens (*P* < 0.01). Furthermore, mutant p53^R172H^ upregulated cavin-1 and promoted invasiveness and metastasis of pancreatic cancer cells *in vitro* and *in vivo*. Finally, combination of mutant p53 and high cavin-1 density indicated the shortest survival for patients with PDAC after resection (*P* < 0.001). Mutant p53-driven upregulation of cavin-1 represents the major mechanism of poor outcome for PDAC patients with the CA19-9 signature after resection, indicating that inhibition of cavin-1 may improve the long-term efficacy of pancreatectomy.

Pancreatic cancer, and more specifically pancreatic ductal adenocarcinoma (PDAC), is the deadliest malignancy of the human digestive system with an estimated 5-year overall survival of about 6%^1^,^2^. Surgical resection of the primary tumor remains the optimal treatment for PDAC. However, surgical outcomes are poor, primarily due to a lack of effective prognosis predicting tools. Some patients are unlikely to benefit from pancreatectomy owing to the presence of occult metastasis at the time of surgery, which is the main reason for poor surgical outcome^3^. Therefore, there is an urgent need to explore potential molecular biomarkers, either from primary tumor tissue or from the peripheral blood, which may predict patient outcome before surgery.

RETRACTED

Some biomarkers have been reported that could predict survival in patients with resectable PDAC, including perioperative serum CA19-9 alterations and major driver-gene mutations^4^,^5^,^6^,^7^,^8^. In our previous study, we identified a preoperative serum signature of CEA^+^/CA125^+^/CA19-9 ≥ 1,000 U/mL that predicted extremely poor outcome after pancreatectomy for patients with PDAC^9^. Patients with this signature were mainly characterized by preoperative CA19-9 ≥ 1,000 U/mL that did not decrease postresection, but the underlying mechanism was unknown.

Four major genes, including *KRAS, TP53, CDKN2A/p16,* and *SMAD4/DPC4*, are the most frequently mutated genes in the landscape of the human PDAC genome as revealed by whole-exome sequencing^10^. Mutations of these driver-genes have been strongly associated with malignant behavior of the tumor and may assist in making an optimal therapeutic selection^6^,^7^,^8^,^11^,^12^,^13^. Notably, serial accumulation of these mutations can also lead to pancreatic carcinogenesis in genetically engineered mouse models^14^. Additionally, it has long been recognized that the serum CA19-9 level reflects the tumor burden in PDAC and could be used to predict patient survival^15^,^16^,^17^. However, it remains ambiguous whether there is a direct correlation between CA19-9 and driver-gene mutations. It is also unclear, which mutation, as well as the downstream mechanism, is mainly responsible for the changes in CA19-9. Thus, our present study aimed to explain the variation in CA19-9 and the response to pancreatectomy from the perspective of genetic alterations.

Caveolin-1 is an essential scaffold protein of caveolae^18^. Cumulative studies have demonstrated that the cavins/caveolin-1 functional axis plays a critical role in the process of caveolae-modulated tumor development^18^,^19^,^20^,^21^,^22^. Our previous study also revealed an indispensable role for polymerase I and transcript release factor (PTRF)/cavin-1, but not cavin-2, -3, and -4, in PDAC progression, where we showed that cavin-1 significantly enhanced caveolin-1-elicited epithelial-mesenchymal-transition (EMT) in pancreatic cells via the activation of the phosphoinositide-3-kinase (PI3K)/Akt signaling pathway^23^. However, the upstream regulatory mechanism is not well understood. Tanase *et al.*^24^ found that overexpression of caveolin-1 correlates with tumor progression biomarkers, such as *TP53* mutation and CA19-9 level, in PDAC, suggesting that specific driver-gene mutations might regulate the cavin-1/caveolin-1 axis. Nonetheless, the specific mutations that drive this regulation have not been elucidated.

RETRACTED

In this study, we found that overexpression of mutant p53, rather than complete loss of p53 expression, was the major genetic alteration in PDAC for patients with preoperative CA19-9 ≥ 1,000 U/mL that did not decrease postresection. Then, we further identified cavin-1 as the only meaningful molecule in the cavins/caveolin-1 axis in the same landscape. Finally, we investigated how mutant p53 regulated cavin-1/caveolin-1, thereby affecting the invasion and metastasis of pancreatic cancer cells.

## Results

### Clinical results and patient outcome

We first performed an analysis of clinicopathological variables and their association with overall survival (OS) and relapse-free survival (RFS) in a training cohort. Patients with a high preoperative serum CA19-9 level, large tumor size, low tumor differentiation, lymph node involvement, microvascular invasion, perineural invasion, and high TNM stage had poorer clinical outcomes after resection of PDAC (all variables: *P* < 0.05 for both OS and RFS, Table 1). Adjuvant chemotherapy prolonged postoperative OS and RFS (*P* < 0.05). Furthermore, the resection method (R0 *vs.* R1) had only borderline significance.

A total of 89 cases with preoperative CA19-9 ≥ 1,000 U/mL were re-evaluated. The median OS and RFS for these patients were dramatically lower than those with CA19-9 < 1,000 U/mL (*n* = 152) (10 *vs.* 20 months for OS, *P* < 0.001; and 6.8 *vs.* 15.5 months for RFS, *P* < 0.001). In subgroup analysis, patients with CA19-9 ≥ 1,000 U/mL that did not decrease postresection had worse prognosis than those with CA19-9 that did decrease postresection (6 *vs.* 11.8 months for OS, *P* < 0.001; and 3.8 *vs.* 8.5 months for RFS, *P* < 0.001; Table 1).

### Overexpression of mutant p53 in PDAC patients with preoperative CA19-9 ≥ 1,000 U/mL that did not decrease postresection

To determine the mutational landscape in the patient cohort, the mutational status of three driver-genes and the expression of normal K-ras protein in PDAC were determined by immunohistochemistry (Supplementary Figure S1). The results showed that mutations in *TP53, CDKN2A/p16,* and *SMAD4/DPC4* occurred at rates of 72%, 41%, and 44%, respectively. As activating overexpression of *KRAS* were near ubiquitous, patients were divided into high or low subgroups according to their sustained expression of K-ras protein. Next, the expression of the driver-genes was classified and analyzed according to the CA19-9 categorization. The *TP53* mutation status was significantly different between the two CA19-9 subgroups, whereas the other two driver-gene mutations had no statistical difference (Supplementary Table S1). Patients with CA19-9 ≥ 1,000 U/mL were more prone to carry *TP53* mutations (*P* < 0.001).

RETRACTED

*TP53* mutation in PDAC includes two subtypes, i.e., the complete loss of p53 protein expression and overexpression of mutant p53, as determined by immunohistochemistry (Fig. 1)^8^. In the 174 cases with *TP53* mutation, 48% (84/174) overexpressed mutant p53. Furthermore, the rate of *TP53* mutation was 100% in patients with preoperative CA19-9 ≥ 1,000 U/mL that did not decrease postresection, while the frequency of mutant p53 overexpression was 89% (24/27, *P* = 0.002) in patients with preoperative CA19-9 ≥ 1,000 U/mL that did decrease postresection (Supplementary Table S2), suggesting that overexpression of mutant p53 is a major player in the mutational landscape of this specific PDAC cohort.

### High expression of cavin-1 in PDAC patients with preoperative CA19-9 ≥ 1,000 U/mL that did not decrease postresection

First, patients were categorized into “high” or “low” groups based on their expression of all of the known critical molecules in the cavins/caveolin-1 axis, and their survival after resection was determined (Table 1). Then, the expression levels of these molecules according to CA19-9 status were evaluated. Compared to patients with CA19-9 < 1,000 U/mL, the expression of caveolin-1 and cavin-1 were significantly higher in patients with CA19-9 ≥ 1,000 U/mL (*P* = 0.011 and *P* < 0.001, respectively), whereas no statistical difference was found for the expression of other molecules, including cavin-2, -3, and -4 (Supplementary Table S1, Fig. 2A–C). Furthermore, the subgroup analysis showed that the expression of cavin-1, but not caveolin-1, was dramatically higher in patients with preoperative CA19-9 ≥ 1,000 U/mL that did not decrease postresection, compared to those with CA19-19 ≥ that did decrease postresection (*P* = 0.010, Supplementary Table S2; Fig. 2D). These results suggest that the cavin-1 may play a role in the mutational p53 landscape in PDAC.

### Correlation between *TP53* mutation and cavin-1 expression in human PDAC

Regardless of CA19-9 categorization, mutant p53 expression was significantly associated with cavin-1 expression in the analysis of the whole population (training cohort: *P* < 0.001, Table 2). Patients with an overexpression of mutant p53 tended to have high cavin-1 expression. Conversely, the complete loss of p53 was not correlated with the cavin-1 expression. In addition, these results could be effectively replicated by using an independent validation cohort (*P* = 0.008).

RETRACTED

### Mutant p53 (*Trp53* ^*R172H*^) upregulates cavin-1 and promotes invasion and metastasis of pancreatic cancer cells

Six common human pancreatic cancer cell lines (Capan-1, SW1990, COLO357, BxPC-3, MiaPaCa-2, and PANC-1) and one human pancreatic duct epithelial cell line (HPDE) were selected and used to determine the protein and mRNA expression of mutant p53, cavin-1, and caveolin-1 by western blot and qRT-PCR, respectively. The MiaPaCa-2 cell line had high expression of mutant p53 and cavin-1, whereas the other cancer cell lines showed only mild expression of both molecules. Furthermore, caveolin-1 was not uniformly expressed (Fig. 3A,B). Next, p53^R172H^-shRNA was transfected into MiaPaCa-2 cells to knockdown the expression of mutant p53. Following transduction, cavin-1 was also downregulated (Fig. 3C,D). Although the proliferation of MiaPaCa-2 was not impaired, the invasiveness markedly decreased, compared with the p53^R172H^-mock-MiaPaCa-2 cells (Fig. 3E–G). Likewise, knockdown of cavin-1 through transduction of cavin-1-shRNA into wild-type MiaPaCa-2 cells achieved the same results as knockdown of mutant p53, while transfection of cavin-1 into the mutant p53 knockdown-MiaPaCa-2 cells reversed and enhanced the invasiveness of the pancreatic cancer cells relative to vector control (Fig. 3C–G). Finally, MiaPaCa-2 cells carrying the abovementioned shRNAs were introduced into nude mice by splenic subcapsular inoculation. Tumor metastatic loci in the liver were visualized by bioluminescence and quantitatively analyzed. The knockdown of mutant p53 or cavin-1 also reduced the metastasis of MiaPaCa-2 cells in the nude mice model, and overexpression of cavin-1 restored this metastatic capability (Fig. 3H,I).

### Combination of mutant p53 and strong cavin-1 expression is associated with the shortest survival for patients with PDAC after resection

In univariate analysis, both mutant p53 and cavin-1 were associated with OS and RFS (*P* < 0.001 for all, Table 1). Patients with an overexpression of mutant p53 and high cavin-1 expression tended to have lymph node involvement, microvascular and perineural invasion, and a high T factor or TNM stage (*P* < 0.05 for all, Table 2), as well as shorter postoperative OS and RFS. Variables showing significance by univariate analysis were adopted when the multivariate Cox proportional hazards regression analysis was performed (Supplementary Table S3). Both overexpression of mutant p53 and high cavin-1 density were independent risk factors for OS (*P* = 0.030 and *P* < 0.001, respectively) and RFS (*P* = 0.002 and *P* < 0.001, respectively). Then, patients were re-divided into three subgroups according to their mutant p53 status and cavin-1 density: group I with non-mutant p53 status and low cavin-1 density (*n* = 130), group II with non-mutant p53 status and high cavin-1 density, or mutant p53 status and low cavin-1 density (*n* = 58), and group III with mutant p53 status and high cavin-1 density (*n* = 53). The estimated median OS was 23, 16, and 8.5 months for groups I, II, and III, respectively (*P* < 0.001, Fig. 4A); the median RFS was 18, 11.2, and 4 months for these same groups, respectively (*P* < 0.001, Fig. 4B). Patients with mutant p53 and strong cavin-1 expression had the shortest survival after resection of PDAC. Furthermore, when performing multivariate analysis, the combination of mutant p53 and strong cavin-1 expression was also an independent prognostic factor for both OS and RFS (*P* < 0.001, Supplementary Table S4). Furthermore, these results could also be validated by using an independent validation cohort (*n* = 78, Fig. 4C,D).

RETRACTED

## Discussion

In the present study, we identified overexpression of mutant p53, rather than complete loss of p53 expression, and high expression of cavin-1 in PDAC patients with a preoperative serum signature of CA19-9 ≥ 1,000 U/mL that did not decrease postresection. Through correlation analysis, we found that overexpression of mutant p53 was significantly associated with high cavin-1 expression in tumor cells. In particular, the combination of the two was associated with the shortest survival for patients with resectable PDAC. Furthermore, we confirmed that mutant p53 (*Trp53*^*R172H*^) promoted the invasion and metastasis of pancreatic cancer cells *in vitro* and *in vivo* via the upregulation of cavin-1 and the enhancement of cavin-1/caveolin-1 signaling.

In pancreatic adenocarcinoma, CA19-9 is recognized as the most important serum tumor biomarker, which fittingly reflects the tumor burden and positively correlates with the malignancy of tumor cells^16^,^26^,^27^,^28^. Moreover, mutations in four major driver-genes, *KRAS, TP53, CDKN2A/p16,* and *SMAD4/DPC4*, are considered to be the impetus of malignant transformation of PDAC^10^,^13^,^14^. Patient subtypes with a higher mutation rate of these genes and their accumulation often have earlier recurrence and a shorter survival after surgery^8^. Thus, we reasonably speculated that the mutations of major genes drive PDAC development and progression, which results in elevated levels of CA19-9. In our previous studies, we found that there was a significant correlation between the driver-gene mutation and the CA19-9 level^28^,^29^, which indirectly supported our hypothesis. However, in this specific cohort of patients with preoperative CA19-9 ≥ 1,000 U/mL that did not decrease postresection, it is unclear, which mutation drives the elevation of CA19-9. In the present study, we identified the aberrant protein expression of mutant p53 as mainly responsible for the phenotypic pattern of CA19-9 in this cohort through immunohistochemically-detected expression of the four driver-genes.

RETRACTED

Mutations of the *TP53* tumor suppressor include two subtypes, complete loss of p53 expression and overexpression of mutant p53, which inactivate wild-type p53 functions and produce “gain-of-function” oncogenic properties, respectively. Here, we showed that patients with overexpression of mutant p53 were prone to develop microvascular invasion, lymph node involvement, and perineural invasion, which contribute to the poor clinical outcome. In previous studies, Morton *et al.* found that mutant p53^R172H^, as compared with genetic loss of p53, specifically drives metastasis and allows cells to circumvent Kras^G12D^-induced growth arrest/senescence in PDAC^30^. Furthermore, Weissmueller *et al.* showed that the sustained expression of the mutant *TP53* allele is necessary to maintain the invasive phenotype of PDAC cells by increasing the expression of cell-autonomous PDGF receptor-β^31^. Thus, it follows that invisible metastatic foci would more likely occur in patients with sustained expression of mutant p53. Once the primary tumor is removed, the residual and premetastatic tumor cells lose their inhibitory factors and are able to proliferate, as confirmed in our previous study^32^, thus producing early recurrence and metastasis. According to this assumption, patients experiencing these phenotypic effects of mutant p53 would most likely be characterized by CA19-9 ≥ 1,000 U/mL that does not decrease postresection. Consequently, this patient population would exhibit a poor response to pancreatectomy.

Increasing evidence gleaned from studies of mutant p53 indicates that it may modulate multiple genes^33^, as does wild-type p53. Nonetheless, whether it can regulate the cavins/caveolin-1 axis and its regulatory targets in pancreatic cancer are poorly understood. An intimate relationship has been shown to exist between p53 and caveolin-1 expression^24^,^34^, but we were unable to identify a similar association between them (data not shown). Intriguingly, we found that both mutant p53 and the essential caveolar component cavin-1 were overexpressed and correlated with one another in this CA19-9 cohort. We also demonstrated that mutant p53 interacted with cavins/caveolin-1 signaling pathway primarily through the regulation of cavin-1. Wild-type p53 has also been reported to mediate the biological function of cavin-1^35^,^36^. This is probably owing to the wild-type p53 exerts its normal cell proliferation-inhibitory function. In summary, our present results, together with results from our previous study^23^, strongly support cavin-1/caveolin-1 signaling as a downstream transcriptional regulator of mutant p53, instead of other gain-of-function activities^33^, which requires further verification.

RETRACTED

Our study had some limitations. Even though it was an effective way to reflect the biological characteristics of CA19-9 from the aspect of genetic mutations, we could not correlate mutation of *TP53* with the generation and secretion of CA19-9 at the DNA/RNA level, because the mechanism of CA19-9 regulation is currently unknown. In addition, although increases in cavin-1 expression were necessary and sufficient to mediate mutant p53 effects in our investigation, mutant p53 exerted cellular effects through the regulation of multiple downstream mediators rather than by modulating a single signaling pathway, which is worth exploring further by transcriptional profiling and functional screening. Nevertheless, our results warrant further clinical investigation of combining mutant p53 status and cavin-1 expression as another indicator for predicting outcome in resectable PDAC, since resection did not benefit those patients whose cancers overexpressed both molecules.

Finally, our findings have important clinical implications. Although surgical resection is still the best method to prolong survival in patients with resectable PDAC^1^, there are a subgroup of patients that do not benefit from pancreatectomy. We previously identified a preoperative serum signature of CEA^+^/CA125^+^/CA19-9 ≥ 1,000 U/mL that was associated with a poor response to surgery, and uncovered a potential mechanism in the present study. Taken together, our results show that mutant p53^R172H^ drives the poor outcome of pancreatic cancer with respect to pancreatectomy by upregulating a critical molecule, cavin-1. Thus, inhibition of cavin-1, either by using small molecule inhibitors or monoclonal antibodies, may improve the long-term efficacy of surgery.

## Methods

### Patient cohort

From January 2009 to December 2014, 657 consecutive patients with pathology-proven PDAC underwent curative resection at our institute using the consensus criteria for resectability^37^,^38^. Of them, 241 cases (training cohort, Table 1) were retrieved from a prospectively collected database (123 Whipple pancreaticoduodenectomies, 115 distal pancreatectomies, and three total pancreatectomies). Entire tumor specimens were collected and preserved under appropriate conditions. Tumors were staged according to the tumor-node-metastasis (TNM) classification system^39^. Patients were followed until April 2015, with a median time of 18.5 months. Overall survival (OS) and recurrence-free survival (RFS) were defined as the interval between the dates of surgery and death or recurrence, respectively. If recurrence was suspected, computerized tomography scanning or magnetic resonance imaging was performed; if recurrence was not diagnosed, patients were censored on the date of death or the last follow-up. The 1-, 3-, and 5-year OS rates were 78%, 33%, and 8%, respectively; the 1-, 3-, and 5-year recurrence rates over the same time intervals were 33%, 71%, and 88%, respectively. Additionally, another independent validation cohort, which contained 78 cases, was also used (40 Whipple pancreaticoduodenectomies, 37 distal pancreatectomies, and one total pancreatectomy). These patients were followed between December 2011 and April 2014, and the median observation time was 12.3 months. This study was approved by the Research Ethics Committees of Fudan University Shanghai Cancer Center, and informed consent was obtained from each patient. The methods were carried out in accordance with the approved guidelines (please see our guidelines using the following link: http://www.nature.com/srep/policies/index.html#experimental-subjects for details).

RETRACTED

### Tissue microarrays (TMAs), immunohistochemistry, and evaluation

The TMA was constructed as described^38^,^40^. Two 1.0 mm diameter tissue cores, drilled from representative areas of each formalin-fixed, paraffin-embedded tumor specimen, were arrayed and constructed into TMAs (Shanghai Biochip Company Ltd., Shanghai, China). Then, four chips for the training cohort and two chips for the validation cohort were prepared.

All of the driver-genes (*KRAS, TP53, CDKN2A/p16,* and *SMAD4/DPC4*) and the critical molecules (cavin-1, -2, -3, -4, and caveolin-1) in the cavins/caveolin-1 axis were screened. Immunohistochemical staining for protein expression of these molecules in the TMA slices (4-μm thick) was performed by a two-step method as described^38^,^41^. The primary and secondary antibodies are listed in the Supplementary Materials and Methods. All slices were stained using the same automation system. Images of five representative fields at ×200 magnification were captured. The density of positive immunostaining in the whole view was measured by a computerized imaging system^38^,^40^,^41^, and the integrated optical density (IOD) for each image was measured using Image-Pro Plus v6.2 software. An identical setting for all images was applied. The results were quantified as IOD/total area^40^.

RETRACTED

X-tile Plots v3.6.1 (Yale University, New Haven, CT) was applied to find an optimal cut-point for each molecule^42^,^43^, and the median value was used as the cut-point for those without an optimal *P* value. Immunohistochemical labeling of three driver-genes (*TP53, CDKN2A/p16,* and *SMAD4/DPC4*) in PDAC accurately reflects their genetic mutational status^8^,^44^, and we adopted this evaluation method. For immunohistochemistry of p53, an antibody that can recognize both wild-type and mutant forms of human p53 protein was utilized. Because *KRAS* is mutated in virtually all PDACs^10^, we used IOD to assess normal K-ras expression and the median value as the cut-point in this study. Accordingly, patients were divided into high- and low-density groups (Supplementary Table S1).

### Cell lines, interventions, and assays

Six common human pancreatic cancer cell lines, including Capan-1, SW1990, COLO357, BxPC-3, MiaPaCa-2, and PANC-1 (American Type Culture Collection, Manassas, VA), with various metastatic potential, were utilized. One human pancreatic duct epithelial cell line, HPDE (Japanese Cancer Research Resources Bank, Tokyo, Japan), was used as negative control. Cells were cultured in complete growth media and used to conduct western blot (WB), quantitative real-time polymerase chain reaction (qRT-PCR), cell transfection (gene knockdown by RNA interference and overexpression), proliferation, and transwell invasion assays, which have been described previously^23^,^32^. The methodological details are given in the Supplementary Methods.

### Nude mouse study

Green fluorescent protein (GFP)-transfected MiaPaCa-2 cells were first established and then used to construct a spleen subcapsular inoculation nude mouse model. Male athymic BALB/c-nu/nu mice of 4–6 weeks of age and weighing about 20 g were used as host animals. Animal care and experimental protocols were approved by the Shanghai Medical Experimental Animal Care Commission, China. The experimental methods were carried out in accordance with the approved guidelines (please see our guidelines using the following link: http://www.nature.com/srep/policies/index.html#experimental-subjects for details). Briefly, approximately 2 × 10^8^ cells, mixed with Matrigel, were inoculated aseptically into the spleen subcapsular of a mouse. After growth for 8 weeks, mice were euthanized and the livers were harvested and evaluated under a fluorescent stereomicroscope^45^.

### Statistical analysis

Statistical analysis was performed with SPSS v18.0 software. Qualitative variables were compared using the Pearson χ^2^ test, and quantitative variables were analyzed with the Student’s *t-*test or Spearman test. Cumulative survival curves were estimated with the Kaplan–Meier method, and the differences between the curves were calculated with the log-rank test. The independent prognostic significance of variables identified with univariate analysis was assessed with Cox proportional hazards regression multivariate analysis. Statistical significance was set at a two-sided *P* value < 0.05.

RETRACTED

## Additional Information

**How to cite this article**: Xiang, J.-F. *et al.* Mutant p53 determines pancreatic cancer poor prognosis to pancreatectomy through upregulation of cavin-1 in patients with preoperative serum CA19-9 ≥1,000 U/mL. *Sci. Rep.* **6**, 19222; doi: 10.1038/srep19222 (2016).

## Supplementary Material

Supplementary Information

## Figures and Tables

**Figure 1:** Images from representative specimens with normal and abnormal immunohistochemical labeling profiles of p53 in pancreatic ductal adenocarcinoma (PDAC). (**A–C**) Sporadic positive nuclear immunolabeling of p53 in ductal and acinar cells of peritumoral normal pancreatic tissue, compared with abnormal expression of p53 in tumor tissue. (**D**) PDAC tissue with a “normal” pattern of p53 immunolabeling compared with normal pancreatic tissue. (**E,F**) An abnormal pattern of p53 immunolabeling^8^, including (**E**) almost complete loss of p53 expression (nuclear immunolabeling in <5% of neoplastic cells) and (**F**) overexpression of mutant p53 (diffuse nuclear accumulation of immunolabeled protein in ≥30% of neoplastic cells), in neoplastic cells of PDAC. The original magnification is shown on each image. *A*, abnormal; *N*, normal.

**Figure 2:** Expression of molecules in the cavins/caveolin-1 axis in pancreatic ductal adenocarcinoma (PDAC). (**A**,**B**) Representative images of low and high cavin-1 expression in PDAC tissue. Cavin-1 was mainly located in the cytoplasm of neoplastic cells, and scattered expression was also seen in the nuclei (×200 magnification). (**C**) The differentially expressed molecules in the cavins/caveolin-1 axis in the training cohort according to the CA19-9 categorization. Compared with patients with CA19-9 < 1,000 U/mL, the levels of cavin-1 and caveolin-1 were significantly higher in patients with CA19-9 ≥ 1,000 U/mL (^*^P < 0.01), whereas no statistical difference was found for cavin-2, -3, and -4. (**D**) Differential expression of cavin-1 and caveolin-1 in subgroups of patients with CA19-9 ≥ 1,000 U/mL. The level of cavin-1, rather than caveolin-1, was dramatically higher in patients with CA19-9 that did not decrease postresection, compared with patients whose CA19-9 did decrease postresection (^*^P = 0.017).

RETRACTED

**Figure 3:** Mutant p53 drives invasiveness and metastasis of pancreatic cancer cells *in vitro* and *in vivo* through the upregulation of cavin-1. (**A**,**B**) Six human pancreatic cancer cell lines and one human pancreatic duct epithelial cell line (HPDE) were used to screen the level of mutant p53, cavin-1 and caveolin-1 protein, and mRNA expression by western blot (WB) and quantitative real-time polymerase chain reaction (qRT-PCR), respectively. (**A**) WB was performed as described^23^. For the detection of p53, an antibody that can only recognize mutant, but not wild-type, p53 was used. (**B**) Levels of mRNA were assessed by qRT-PCR and normalized to the corresponding internal β-actin signal (ΔCT); the relative gene expression values were expressed as 2^−ΔCT^ 32. ^*^P < 0.05, compared with each group. (**C**,**D**) Expression of mutant p53, cavin-1, and caveolin-1 after shRNA treatment was validated by WB and qRT-PCR. ^*,#^*P* < 0.05, compared with the wild-type and mock group; ^**^P < 0.05, compared with the shp53-mock group. (**E**) A Cell Counting Kit-8 was used to assay cell proliferation. No significant difference was found among groups. OD, optical density. (**F**,**G**) Cell invasiveness was assayed in Matrigel-coated Transwell Invasion Chambers. Cell cultures were incubated for 72 h, and the cells that passed through the membranes were counted (at ×200 magnification). ^*^P < 0.01, compared with the mock group; ^#^*P* < 0.05, compared with the shp53-mock group. (**H**,**I**) Representative bioluminescence and hematoxylin-eosin (HE) images of tumor metastatic foci in nude mouse livers (*n* = 6). The morphology was detected in general, and the number was counted. ^*^P < 0.05, compared with the mock group; ^#^*P* < 0.05, compared with the shp53-mock group.

**Figure 4:** Cumulative (**A**) overall and (**B**) recurrence-free survival curves of the combination of intratumoral mutant p53 and cavin-1 expression, and (**C**, **D**) their validation. Patients with the combination of mutant p53 status and strong cavin-1 expression (group III) had the shortest survival after resection of PDAC.

**Table 1:** Univariate analyses of variables for survival and recurrence in the training cohort (*n* = 241).

Variables	No. of patients (%)	Overall survival		Recurrence-free survival	
		Median* (Months)	Log-rank (*P* value)	Median* (Months)	Log-rank (*P* value)
Gender			0.813		0.626
Female	92 (38)	16		12	
Male	149 (62)	18		13	
Age, years					
Mean ± SD	60.95 ± 9.74				
Median (Range)	62 (35–79)				
Preoperative CA19-9, U/mL			<0.001		<0.001
<1000	152 (63)	20		15.5	
≥1000	89 (37)	10		6.8	
Decreased postresection	62 (70)	11.8	<0.001	8.5	<0.001
Did not decrease postresection	27 (30)	6		3.8	
Tumor size, cm			<0.001		0.001
≤2	107 (44)	20		13	
>2	134 (56)	16		12	
Tumor location			0.989		0.312
Head	130 (54)	17		12	
Body/tail	111 (46)	18		13	
Tumor differentiation			<0.001		0.002
Low (Stage III–IV)	132 (55)	16.5		12	
High (Stage I–II)	109 (45)	18		13	
Lymph node involvement			<0.001		<0.001
No	112 (46)	19		16	
Yes	129 (54)	16.5		12	
Microvascular invasion			0.032		<0.001
No	177 (73)	18		15	
Yes	64 (27)	16.1		11	
Perineural invasion			0.001		0.005
No	83 (34)	23		16.5	
Yes	158 (66)	16		12	
T factor (UICC)			<0.001		<0.001
T1/T2	87 (36)	19		14	
T3	154 (64)	16.5		12	
TNM stage (UICC)			<0.001		<0.001
IB	38 (16)	26		22	
IIA	74 (31)	19		13	
IIB	129 (53)	17		12	
Margin status			0.076		0.095
R0	168 (70)	18		13.3	
R1	73 (30)	14		11	
Adjuvant chemotherapy			0.041		0.014
No	78 (32)	16.5		12	
Yes	163 (68)	17.2		13	
K-ras density			0.271		0.344
Low	120 (50)	17.8		12	
High	121 (50)	17		13	
p53 staining			0.001		0.002
Normal	67 (28)	20		15	
Abnormal	174 (72)	16.5		12	
Mutant p53	84 (35)	10.5	<0.001	6.2	<0.001
Non-mutant p53	157 (65)	20		15.5	
p16 staining			0.019		0.041
Positive/intact	142 (59)	18		12.5	
Negative/loss	99 (41)	16.5		12	
Smad4 staining			<0.001		<0.001
Positive/intact	135 (56)	20		15	
Negative/loss	106 (44)	14		11.1	
Cavin-1 density			<0.001		<0.001
Low	161 (67)	20		15.5	
High	80 (33)	11		7.8	
Cavin-2 density			0.145		0.094
Low	120 (50)	16.1		12	
High	121 (50)	18		13	
Cavin-3 density			0.579		0.825
Low	120 (50)	18		13	
High	121 (50)	17		12	
Cavin-4 density			0.172		0.223
Low	120 (50)	17.2		12	
High	121 (50)	17		12.5	
Caveolin-1 density			<0.001		<0.001
Low	126 (52)	23		16	
High	115 (48)	13		11	
Combined mutant p53 and cavin-1			<0.001		<0.001
Low risk	130 (54)	23		18	
Moderate risk	58 (24)	16		11.2	
High risk	53 (22)	8.5		4	

Abbreviations: SD, standard deviation; UICC, Union for International Cancer Control; TNM, tumor-node-metastasis.

^*^Estimated median overall survival and recurrence-free survival by the log-rank test.

RETRACTED

**Table 2:** Correlations between the overexpression of mutant p53 and cavin-1 expression with clinicopathological parameters in the training cohort.

Variables	p53 staining			Cavin-1 density		
	Mutant (*n* = 84) No. (%)	Non-mutant (*n* = 157) No. (%)	*P* value	Low (*n* = 161) No. (%)	High (*n* = 80) No. (%)	*P* value
Gender			0.985			0.879
Female	32 (38)	60 (38)		62 (39)	30 (38)	
Male	52 (62)	97 (62)		99 (61)	50 (62)	
Age, years			0.150			0.676
≤60	32 (38)	75 (48)		73 (45)	34 (43)	
>60	52 (62)	82 (52)		88 (55)	46 (57)	
Preoperative CA19-9, U/mL			<0.001			<0.001
<1000	26 (31)	126 (80)		123 (76)	29 (36)	
≥1000	58 (69)	31 (20)		38 (24)	51 (64)	
Tumor size, cm			0.002			0.676
≤2	26 (31)	81 (52)		73 (45)	34 (43)	
>2	58 (69)	76 (48)		88 (55)	46 (57)	
Tumor location			0.242			0.966
Head	41 (49)	89 (57)		87 (54)	43 (54)	
Body/tail	43 (51)	68 (43)		74 (46)	37 (46)	
Tumor differentiation			0.104			0.154
Low (Stage III–IV)	52 (62)	80 (51)		83 (52)	49 (61)	
High (Stage I–II)	32 (38)	77 (49)		78 (48)	31 (39)	
Lymph node involvement			0.001			0.009
No	24 (29)	80 (51)		79 (49)	25 (31)	
Yes	60 (71)	77 (49)		82 (51)	55 (69)	
Microvascular invasion			<0.001			<0.001
No	38 (45)	139 (88)		140 (87)	37 (46)	
Yes	46 (55)	18 (12)		21 (13)	43 (54)	
Perineural invasion			0.024			0.030
No	21 (25)	62 (40)		63 (39)	20 (25)	
Yes	63 (75)	95 (60)		98 (61)	60 (75)	
T factor (UICC)			0.009			0.011
T1/T2	21 (25)	66 (42)		67 (42)	20 (25)	
T3	63 (75)	91 (58)		94 (58)	60 (75)	
TNM stage (UICC)			0.046			0.038
IB	7 (8)	31 (20)		32 (20)	6 (8)	
IIA	31 (37)	43 (27)		45 (28)	29 (36)	
IIB	46 (55)	83 (53)		84 (52)	45 (56)	
Cavin-1 density			<0.001			—
Low	31 (37)	130 (83)		—	—	
High	53 (63)	27 (17)		—	—	

Abbreviations: UICC, Union for International Cancer Control; TNM, tumor–node–metastasis.

## References

[b1] RyanD. P., HongT. S. & BardeesyN. Pancreatic adenocarcinoma. N Engl J Med 371, 1039–1049 (2014).2520776710.1056/NEJMra1404198

[b2] DeSantisC. E. *et al.* Cancer treatment and survivorship statistics, 2014. CA Cancer J Clin 64, 252–271 (2014).2489045110.3322/caac.21235

[b3] HartwigW., WernerJ., JagerD., DebusJ. & BuchlerM. W. Improvement of surgical results for pancreatic cancer. Lancet Oncol 14, e476–485 (2013).2407987510.1016/S1470-2045(13)70172-4

[b4] FerroneC. R. *et al.* Perioperative CA19-9 levels can predict stage and survival in patients with resectable pancreatic adenocarcinoma. J Clin Oncol 24, 2897–2902 (2006).1678292910.1200/JCO.2005.05.3934PMC3817569

[b5] TakahashiH. *et al.* Serum CA19-9 alterations during preoperative gemcitabine-based chemoradiation therapy for resectable invasive ductal carcinoma of the pancreas as an indicator for therapeutic selection and survival. Ann Surg 251, 461–469 (2010).2013431510.1097/SLA.0b013e3181cc90a3

[b6] BiankinA. V. *et al.* DPC4/Smad4 expression and outcome in pancreatic ductal adenocarcinoma. J Clin Oncol 20, 4531–4542 (2002).1245410910.1200/JCO.2002.12.063

[b7] Iacobuzio-DonahueC. A. *et al.* DPC4 gene status of the primary carcinoma correlates with patterns of failure in patients with pancreatic cancer. J Clin Oncol 27, 1806–1813 (2009).1927371010.1200/JCO.2008.17.7188PMC2668706

[b8] OshimaM. *et al.* Immunohistochemically detected expression of 3 major genes (CDKN2A/p16, TP53, and SMAD4/DPC4) strongly predicts survival in patients with resectable pancreatic cancer. Ann Surg 258, 336–346 (2013).2347056810.1097/SLA.0b013e3182827a65

RETRACTED

[b9] LiuL. *et al.* A preoperative serum signature of CEA+/CA125+/CA19-9>/=1000 U/mL indicates poor outcome to pancreatectomy for pancreatic cancer. Int J Cancer 136, 2216–2227 (2015).2527394710.1002/ijc.29242

[b10] JonesS. *et al.* Core signaling pathways in human pancreatic cancers revealed by global genomic analyses. Science 321, 1801–1806 (2008).1877239710.1126/science.1164368PMC2848990

[b11] BlackfordA. *et al.* SMAD4 gene mutations are associated with poor prognosis in pancreatic cancer. Clin Cancer Res 15, 4674–4679 (2009).1958415110.1158/1078-0432.CCR-09-0227PMC2819274

[b12] YachidaS. Novel therapeutic approaches in pancreatic cancer based on genomic alterations. Curr Pharm Des 18, 2452–2463 (2012).2237249710.2174/13816128112092452

[b13] WaddellN. *et al.* Whole genomes redefine the mutational landscape of pancreatic cancer. Nature 518, 495–501 (2015).2571966610.1038/nature14169PMC4523082

[b14] HingoraniS. R. *et al.* Trp53R172H and KrasG12D cooperate to promote chromosomal instability and widely metastatic pancreatic ductal adenocarcinoma in mice. Cancer Cell 7, 469–483 (2005).1589426710.1016/j.ccr.2005.04.023

[b15] HumphrisJ. L. *et al.* The prognostic and predictive value of serum CA19.9 in pancreatic cancer. Ann Oncol 23, 1713–1722 (2012).2224189910.1093/annonc/mdr561PMC3387824

[b16] BalzanoG. & Di CarloV. Is CA 19-9 useful in the management of pancreatic cancer? Lancet Oncol 9, 89–91 (2008).1823784710.1016/S1470-2045(08)70011-1

[b17] HataS. *et al.* Prognostic impact of postoperative serum CA 19-9 levels in patients with resectable pancreatic cancer. Ann Surg Oncol 19, 636–641 (2012).2186336010.1245/s10434-011-2020-9

[b18] GoetzJ. G., LajoieP., WisemanS. M. & NabiI. R. Caveolin-1 in tumor progression: the good, the bad and the ugly. Cancer Metastasis Rev 27, 715–735 (2008).1850639610.1007/s10555-008-9160-9

[b19] HillM. M. *et al.* PTRF-Cavin, a conserved cytoplasmic protein required for caveola formation and function. Cell 132, 113–124 (2008).1819122510.1016/j.cell.2007.11.042PMC2265257

[b20] HansenC. G., BrightN. A., HowardG. & NicholsB. J. SDPR induces membrane curvature and functions in the formation of caveolae. Nat Cell Biol 11, 807–814 (2009).1952593910.1038/ncb1887PMC2712677

[b21] McMahonK. A. *et al.* SRBC/cavin-3 is a caveolin adapter protein that regulates caveolae function. EMBO J 28, 1001–1015 (2009).1926256410.1038/emboj.2009.46PMC2683698

[b22] BastianiM. *et al.* MURC/Cavin-4 and cavin family members form tissue-specific caveolar complexes. J Cell Biol 185, 1259–1273 (2009).1954624210.1083/jcb.200903053PMC2712963

RETRACTED

[b23] LiuL. *et al.* Cavin-1 is essential for the tumor-promoting effect of caveolin-1 and enhances its prognostic potency in pancreatic cancer. Oncogene 33, 2728–2736 (2014).2377085710.1038/onc.2013.223

[b24] TanaseC. P. *et al.* Caveolin-1 overexpression correlates with tumour progression markers in pancreatic ductal adenocarcinoma. J Mol Histol 40, 23–29 (2009).1916006410.1007/s10735-008-9209-7

[b25] NenutilR. *et al.* Discriminating functional and non-functional p53 in human tumours by p53 and MDM2 immunohistochemistry. J Pathol 207, 251–259 (2005).1616100510.1002/path.1838

[b26] LockerG. Y. *et al.* ASCO 2006 update of recommendations for the use of tumor markers in gastrointestinal cancer. J Clin Oncol 24, 5313–5327 (2006).1706067610.1200/JCO.2006.08.2644

[b27] PorukK. E. *et al.* The clinical utility of CA 19-9 in pancreatic adenocarcinoma: diagnostic and prognostic updates. Curr Mol Med 13, 340–351 (2013).2333100610.2174/1566524011313030003PMC4419808

[b28] XuH. X. *et al.* Metabolic tumour burden assessed by (1)(8)F-FDG PET/CT associated with serum CA19-9 predicts pancreatic cancer outcome after resection. Eur J Nucl Med Mol Imaging 41, 1093–1102 (2014).2452279710.1007/s00259-014-2688-8

[b29] ShiS. *et al.* Metabolic tumor burden is associated with major oncogenomic alterations and serum tumor markers in patients with resected pancreatic cancer. Cancer Lett 360, 227–233 (2015).2568788310.1016/j.canlet.2015.02.014

[b30] MortonJ. P. *et al.* Mutant p53 drives metastasis and overcomes growth arrest/senescence in pancreatic cancer. Proc Natl Acad Sci USA 107, 246–251 (2010).2001872110.1073/pnas.0908428107PMC2806749

[b31] WeissmuellerS. *et al.* Mutant p53 drives pancreatic cancer metastasis through cell-autonomous PDGF receptor beta signaling. Cell 157, 382–394 (2014).2472540510.1016/j.cell.2014.01.066PMC4001090

[b32] WangW. Q. *et al.* Tanshinone IIA inhibits metastasis after palliative resection of hepatocellular carcinoma and prolongs survival in part via vascular normalization. J Hematol Oncol 5, 69 (2012).2313716510.1186/1756-8722-5-69PMC3506473

[b33] Freed-PastorW. A. & PrivesC. Mutant p53: one name, many proteins. Genes Dev 26, 1268–1286 (2012).2271386810.1101/gad.190678.112PMC3387655

[b34] LeeS. H. *et al.* Extracellular p53 fragment re-enters K-Ras mutated cells through the caveolin-1 dependent early endosomal system. Oncotarget 4, 2523–2531 (2013).2434411410.18632/oncotarget.1550PMC3926846

[b35] BaiL. *et al.* Regulation of cellular senescence by the essential caveolar component PTRF/Cavin-1. Cell Res 21, 1088–1101 (2011).2144510010.1038/cr.2011.56PMC3193497

[b36] VolonteD. & GalbiatiF. Polymerase I and transcript release factor (PTRF)/cavin-1 is a novel regulator of stress-induced premature senescence. J Biol Chem 286, 28657–28661 (2011).2170533710.1074/jbc.C111.235119PMC3190672

RETRACTED

[b37] LiuC. *et al.* Pancreatic stump-closed pancreaticojejunostomy can be performed safely in normal soft pancreas cases. J Surg Res 172, e11–17 (2012).2207984810.1016/j.jss.2011.09.002

[b38] WangW. Q. *et al.* Intratumoral alpha-SMA enhances the prognostic potency of CD34 associated with maintenance of microvessel integrity in hepatocellular carcinoma and pancreatic cancer. PLoS One 8, e71189 (2013).2394071510.1371/journal.pone.0071189PMC3734294

[b39] EdgeS. B. *et al.* AJCC cancer staging manual (7th ed.). New York, Springer (2010).

[b40] ZhuX. D. *et al.* High expression of macrophage colony-stimulating factor in peritumoral liver tissue is associated with poor survival after curative resection of hepatocellular carcinoma. J Clin Oncol 26, 2707–2716 (2008).1850918310.1200/JCO.2007.15.6521

[b41] WangW. Q. *et al.* The combination of HTATIP2 expression and microvessel density predicts converse survival of hepatocellular carcinoma with or without sorafenib. Oncotarget 5, 3895–3906 (2014).2500831510.18632/oncotarget.2019PMC4116529

[b42] CampR. L., Dolled-FilhartM. & RimmD. L. X-tile: a new bio-informatics tool for biomarker assessment and outcome-based cut-point optimization. Clin Cancer Res 10, 7252–7259 (2004).1553409910.1158/1078-0432.CCR-04-0713

[b43] JiaJ. B. *et al.* High expression of macrophage colony-stimulating factor-1 receptor in peritumoral liver tissue is associated with poor outcome in hepatocellular carcinoma after curative resection. Oncologist 15, 732–743 (2010).2055142910.1634/theoncologist.2009-0170PMC3228006

[b44] YachidaS. *et al.* Clinical significance of the genetic landscape of pancreatic cancer and implications for identification of potential long-term survivors. Clin Cancer Res 18, 6339–6347 (2012).2299141410.1158/1078-0432.CCR-12-1215PMC3500447

[b45] ZhuX. D. *et al.* Antiangiogenic therapy promoted metastasis of hepatocellular carcinoma by suppressing host-derived interleukin-12b in mouse models. Angiogenesis 16, 809–820 (2013).2371600010.1007/s10456-013-9357-6

